# Application of LSTM Neural Network Technology Embedded in English Intelligent Translation

This article has been retracted.

**DOI:** 10.1155/2022/1085577

**Published:** 2022-09-27

**Authors:** Yifang Yang

**Affiliations:** School of Humanities, Hunan City University, Yiyang, Hunan 413000, China

## Abstract

With the rapid development of computer technology, the loss of long-distance information in the transmission process is a prominent problem faced by English machine translation. The self-attention mechanism is combined with convolutional neural network (CNN) and long-term and short-term memory network (LSTM). An English intelligent translation model based on LSTM-SA is proposed, and the performance of this model is compared with other deep neural network models. The study adds SA to the LSTM neural network model and constructs the English translation model of LSTM-SA attention embedding. Compared with other deep learning algorithms such as 3RNN and GRU, the LSTM-SA neural network algorithm has faster convergence speed and lower loss value, and the loss value is finally stable at about 8.6. Under the three values of adaptability, the accuracy of LSTM-SA neural network structure is higher than that of LSTM, and when the adaptability is 1, the accuracy of LSTM-SA neural network improved the fastest, with an accuracy of nearly 20%. Compared with other deep learning algorithms, the LSTM-SA neural network algorithm has a better translation level map under the three hidden layers. The proposed LSTM-SA model can better carry out English intelligent translation, enhance the representation of source language context information, and improve the performance and quality of English machine translation model.

## 1. Introduction

Computer science and technology and artificial intelligence are inextricably linked. The disciplines related to artificial intelligence include computer, software programming, and other related disciplines. Colleges and universities that offer artificial intelligence related disciplines may offer them in mechanical engineering, electrical engineering, information engineering, automation, and other related disciplines. Because of its high speed and low cost, machine translation is regarded as an important means to overcome communication barriers between different languages. In recent years, with the development of deep learning, neural machine translation based on “encoder-decoder” architecture has become a mainstream machine translation research method. However, due to the limited size of the vocabulary and the imperfect coverage mechanism, there are many problems in neural machine translation, such as unknown words, over translation, and missing translation. With the continuous development and maturity of artificial intelligence technology and computer technology, intelligent translation is gradually replacing human translation and gradually occupying a greater proportion in the field of translation. At present, common machine translation mainly includes neural network, statistics, examples, and rules [1]. Among them, the machine translation model of neural network can avoid the feature design problem of high-dimensional complex data by constructing neural network classifier when dealing with high-dimensional data and greatly improves the expression ability of the model. The model has gradually become the most widely used language translation model [2]. The most effective and widely used neural network language translation models are GRU attention, recurrent neural network (RNN), long short-term memory (LSTM) neural network, etc. They have been widely used in the field of English machine translation [3]. Most mathematicians at home and abroad have analyzed English machine translation through neural networks with different structures, and then completed intelligent standardized English machine translation [4]. However, the current English machine translation model based on neural network structure has less obvious translation effect due to the problem of information loss in the process of long-distance information transmission. By adding the self-attention (SA) mechanism to LSTM neural network model, an English translation model of LSTM attention embedding is constructed. LSTM, like RNNs, can handle time series tasks better than CNN. At the same time, LSTM solves the problem of long-term dependence of RNN and alleviates the problem of “gradient disappearance” caused by reverse propagation of RNN during training. The model structure of LSTM itself is relatively complex, and the training is more time-consuming than CNN. In addition, the characteristics of RNN networks determine that they cannot process data in parallel. Furthermore, LSTM alleviates the long-term dependence of RNN to a certain extent. But for longer sequence data, LSTM is also very difficult.

The innovative contribution of this research lies in the application of LSTM-SA combinatorial model to English translation. Adding SA to the LSTM neural network model improves the ability of the model to capture medium and long-distance dependent features. Since any two data can be calculated and connected by the weight matrix of the self-focusing model, the relationship between distance-related features is shortened. It can not only avoid the problem that the English input sequence and the model cannot match completely but also improve the translation effect to a great extent. The convolution model of LSTM has a better ability to extract the mutual attention of time series and the internal relationship of time series. LSTM neural network can extract time series data. Compared with other neural network models, LSTM neural network has strong advantages.

This paper is divided into five parts.  Section 1 expounds that computer science and technology are inseparable from artificial intelligence. Intelligent translation is gradually replacing manual translation.  Section 2 analyzes the research status of LSTM neural network and English intelligent translation.  Section 3 analyzes the construction of English intelligent translation model through SA and LSTM. At the same time, the English intelligent translation model of LSTM-SA is expounded.  Section 4 summarizes the application effect analysis of English intelligent translation. The motion detection results of LSTM-SA and LSTM neural network structure show that LSTM-SA neural network is the best in the adaptability of neural network. The LSTM-SA neural network algorithm has faster convergence speed and more stable loss value.  Section 5 evaluates the research results and puts forward the shortcomings and future prospects of the research.

## 2. Related Works

In order to evaluate how the complexity of climate model affects the prediction skills of neural network, Scher and Messori took atmospheric circulation models with different complexity as the research background and completed the prediction of climate and weather with the help of deep neural network. The simulation results show that it is still challenging to use neural network to reproduce the climate of atmospheric circulation model including seasonal cycle [5]. Gao analyzed the development and reform of College English teaching mode under artificial intelligence. The improved contents include the organizational form of teaching, the presentation form of teaching resources, and the form of teaching evaluation. The research confirmed that artificial intelligence assisted language learning is very important for the improvement of English teaching mode [2]. Ernawati et al. used multiple intelligence to evaluate and identify students' intelligence and obtained effective English teaching methods for children. The example analysis results show that multiple intelligences evaluation can help teachers find students' interests and guide them to establish some learning activities to attract them to learn English [6]. Aiming at the integration development trend of college English culture teaching mode and modern information technology, Meng-yue et al. have constructed an intelligent auxiliary system. The research results verify that modern information technology can innovate and develop college English culture teaching [7]. Takahashi and Tanaka-Ishii used the most advanced computational language model, and combined with the selected information theory measurement and computational language model, the computational language model captures the changes of language and discusses the benefits and limitations. The research results enrich the data-driven theory [8]. Goldstein et al. designed a recurrent graph neural network structure and applied it to grape vine pruning. The simulation results show that the automatic pruning effect of grape vine is good [9]. Li and Wang used the improved positioning method of deep belief network to carry out real-time position control and state recognition for online learning students. The results show that the recognition effect of the student online learning recognition model based on artificial intelligence is good [10].

Chen and Joo proposed a new method for estimating the three-dimensional direction of arrival of electromagnetic signals using convolution neural network in Gaussian and non-Gaussian noise environment. Through infinite norm normalization, pulse outliers can be effectively suppressed, so as to provide appropriate input characteristics for neural network. The simulation results show that in Gaussian and non-Gaussian noise environment, this method is superior and effective in the calculation speed and accuracy of 1D direction of arrival and 3D direction of arrival estimation, and the signal monitoring network can also effectively control the output of the neural network [11]. On the premise that Chakrabarty and Habets clearly know that the sound source location method of supervised learning is data-driven and robust to adverse acoustic environment, they proposed a supervised learning method based on convolutional neural network to estimate the direction of arrival of multiple speakers. The simulated and measured acoustic impulse response evaluation experiments showed the ability of the proposed method to adapt to unknown acoustic conditions and its robustness to unknown noise types and the ability to accurately locate the speaker in a dynamic acoustic scene with a varying number of sources [12]. O'Toole et al. designed a convolutional neural network model based on the sky image, which uses the sky image to predict the global horizontal irradiance one hour ago without numerical measurement and additional feature engineering. The numerical results of six-year data show that the normalized root mean square error is 8.85%, and the prediction skill score is 25.14%, which shows its superiority under various weather conditions [13]. Zheng et al. proposed a hybrid depth convolution neural network model and applied it to solar flare prediction. After the model is verified and trained, the results showed that some key features automatically extracted by our model may not have been mined before and may provide important clues for the study of flare mechanism [14].

From the above research results, it can be concluded that the neural network structure has been widely used in image, computer vision, speech recognition, motion detection, image classification, and so on. However, there are relatively few studies on English intelligent translation, and the relevant research results have not obtained satisfactory results. This paper analyzes English intelligent translation by adding the attention mechanism to the LSTM neural network model in order to provide new research ideas for English intelligent machine translation.

## 3. English Intelligent Translation Model of LSMT-SA

### 3.1. LSMT Neural Network Algorithm

The LSTM neural network structure introduces three logical structures, input gate, output gate, and forgetting gate, on the basis of classical cyclic neural network. The structural diagram is shown in Figure 1. In the LSTM network structure, the input gate, output gate, and forgetting gate use *i*, *o*, and *f* respectively, and the memory unit is *C*, the input data is *X*, and the implicit state is *H*. The forgetting gate clears all the less important information in the cell state. Its input includes the cell state of the specific time step *x*^*t*^ and the upper hidden layer *h*^(*t* − 1)^. The control function determines whether the information is cleared or retained [15]. Finally, the value range of vector *f*^(*t*)^ of the output unit state is [0, 1]. If the value is 1, the input value will be retained as a whole. If the value is 0, the value will be deleted as a whole [16]. Input refers to determining whether the information is added to the cell state for data update, using the SIGMOID function to delete the information of *x*^*t*^ and *h*^(*t* − 1)^, then calculating the current input cell state, and establishing the postselection vector through the tach function, with the value range of [−1, 1], and finally calculating the cell state *c*^(*t*)^ at the current time. This value is multiplied by the cell state *c*^(*t* − 1)^ at the previous time and the forgetting gate, and then added with *c*′^(*t*)^. It is finally multiplied by input gate *i*^(*t*)^ [17].

The output gate is to select the valuable unit state to be presented for output. Its specific implementation process includes two steps. Firstly, a filter *o*^(*t*)^ is obtained by using *x*^*t*^ and *h*^(*t* − 1)^, and then the tach function is selected to compress the value of the unit state vector to [−1, 1]. At the same time, the result is obtained by multiplying the vector, and *o*^(*t*)^ is used as the judgment basis of hidden information *h*^(*t*)^. The algorithm training process first calculates the error of the last layer, then updates the parameters through the gradient descent algorithm, and then passes forward layer by layer until all parameters are updated [18]. Many geometric and topological information in vector graphics must be protected accurately. Otherwise, when the products are designed according to the drawings, minor changes in the drawings may cause the products designed to be unqualified. Therefore, it is more difficult to hide information than the normal still images, audio, and video. Some existing information hiding techniques and secret information detection techniques cannot be directly applied to vector graphics. In the long-term and short-term memory network, there are eight groups of parameters to be learned, including forgetting gate, input gate, output gate, and the weight matrix and bias term of the unit state. The calculation methods of the weight matrix are different in the two directions of back propagation [19].

The specific steps of LSTM neural network model are as follows: firstly, determine the neuron forgetting information, assuming that the batch data with the number of samples contained in time *t* is *n* and *x*, *X*_*t*_ is the vector, *h* refers to the length of the hidden layer, *H*_*t*_ refers to the state of the hidden layer at time *t*, and the state of the hidden layer at the previous time is represented by *H*_*t*−1_. The expression of forgetting gate at time *t* is

(1) $$\begin{array}{c} f_{t}=\sigma \left(X_{t}W_{xf}+H_{t-1}W_{hf}+b_{f}\right)\text{.} \end{array}$$

In formula (1), *σ* refers to sigmoid function, *W*_*f*_ refers to learnable weight parameters, and *b*_*f*_ refers to offset vector parameters. The data operation method of broadcasting is the process of addition.

Secondly, determine the information to be saved by the neural unit. The updated value is preliminarily determined through the sigmoid function network layer, and the calculation expression is

(2) $$\begin{array}{c} i_{t}=\sigma \left(X_{t}W_{xi}+H_{t-1}W_{hi}+b_{i}\right)\text{.} \end{array}$$

In equation (2), *W*_*i*_ refers to the weight of the update door, and *b*_*i*_ refers to the offset of the update door. The candidate values are generated through the hyperbolic tangent function tach layer, and the calculation expression is

(3) $$\begin{array}{c} {\bar{C}}_{t}=\tanh\;\left(X_{t}W_{xc}+H_{t-1}W_{hc}+b_{c}\right)\text{.} \end{array}$$

Next, update the memory status. The state is updated by point multiplication operation, and the output gate and forgetting gate are used to control the flow of information. Finally, the updated state is obtained. The calculation formula is

(4) $$\begin{array}{c} C_{t}=f_{t}\Theta \;\tanh\left(C_{t}\right)\text{.} \end{array}$$

From equation (4), when the forgetting gate approaches 1 and the input gate approaches 0, then the memory unit in the old state will be saved to the current time. LSTM network can handle the phenomenon of gradient disappearance in the circulating nerve [20].

Finally, the memory unit of the output state of the output gate is determined by the sigmoid function:

(5) $$\begin{array}{c} O_{t}=\sigma \left(X_{t}W_{xo}+H_{t-1}W_{ho}+b_{o}\right)\text{.} \end{array}$$

In equation (5), *W*_*o*_ refers to the weight of the output gate, and *b*_*o*_ refers to the offset of the output gate.

The calculation formula of hidden layer state 4 at time 3 is

(6) $$\begin{array}{c} H_{t}=O_{t}\Theta \;\tanh\left(C_{t}\right)\text{.} \end{array}$$

### 3.2. SA Model

SA is a model that can simulate the attention activity of the human brain. The model can input and calculate the attention of a key point, and calculate the influence of the key point output model. The sequence to sequence (seq2seq) model is a special recurrent neural network architecture. It is usually used (but not limited to) to solve complex language problems, such as machine translation, question answering, creating chat robots, and text summarization. Some applications that consider seq2seq is the best solution. The model can be used as a solution to any sequence-based problem, especially for problems with different input and output sizes and categories. The sequence to sequence (seq2seq) model is a model that can solve the problems related to machine translation. It is mainly derived from the structure of RNN model and includes two parts: encoder and decoder. The structure of encoding and decoding has a large degree of freedom. The same type and different types of neural network models can be used. At present, RNN or LSTM models are widely used [21]. In RNN, the state of the neuron is the state of the previous neuron, and the input information *X* of the current neuron are used as the calculation input as

(7) $$\begin{array}{c} o_{t}=f\left(o_{t-1},x_{t}\right)\text{.} \end{array}$$

In the encoding process, the hidden layer state *o*_*t*_ of the last input is regarded as a semantic vector, and all hidden layer states of the input sequence can also be changed nonlinearly to obtain a semantic vector *C*. At the same time, *T* is the number of words in the input sequence as

(8) $$\begin{array}{c} \left\{\begin{array}{c} C=o_{T_{x}},\\ C=q\left(o_{1},o_{2},o_{3},...,o_{T_{x}}\right)\text{.} \end{array}\right. \end{array}$$

In the decoding process, the semantic vector is converted into a specified length sequence. The next output word can be predicted through semantic vector *C* and output sequence *o*_1_, *o*_2_, *o*_3_, ..., *o*_*t*_ is

(9) $$\begin{array}{c} o_{t}=argmaxP\left(o_{t}\right)=\prod_{t=1}^{T}p\left(o_{t}\left|\left\{o_{1},o_{2},...,o_{t-1}\right\},C\right.\right)\\ =g\left(\left\{o_{1},o_{2},...,o_{t-1}\right\},C\right)\text{.} \end{array}$$

When the seq2seq model has only a fixed length semantic vector *C* between the encoder and the decoder, the sequence information is processed into a fixed length vector by the encoder, and the model will have disadvantages such as long-distance dependence [22]. Therefore, SA is introduced. Its main principle is to simulate the processing ability of human brain information, so that when paying attention to something, we can focus on a key part of the thing and find out more useful information. The attention mechanism is usually combined with seq2seq, which can be applied to coding and decoding modules. The basic structure of the attention mechanism is shown in Figure 2.

When attention is applied in the decoding module of the seq2seq model, the conditional probability of the decoding module through the *X* prediction output is calculated as

(10) $$\begin{array}{c} p\left(y_{t}\left|\left\{y_{1},y_{2},...,y_{t-1}\right\},X\right.\right)=g\left(y_{t-1},s_{i},c_{i}\right)\text{.} \end{array}$$

In equation (10), *s*_*i*_ represents the hidden layer state at time *t* during decoding, and its calculation is

(11) $$\begin{array}{c} s_{i}=f\left(s_{i-1},y_{i-1},c_{i}\right)\text{.} \end{array}$$

The language vector *c*_*i*_ corresponding to each target output value *o*_*t*_ will affect the conditional probability, and *c*_*i*_ is obtained by adding the hidden layer vector sequence (*o*_1_, *o*_2_, *o*_3_, ..., *o*_*T*_*x*__) in the decoding module according to the weight by

(12) $$\begin{array}{c} c_{i}=\prod_{j=1}^{T_{x}}\alpha_{ij}o_{j}\text{.} \end{array}$$

Language vector *c*_*i*_ is inconsistent in the attention distribution of the *j* output. This is an information screening method that can further alleviate the long-term dependency problem in LSTM and GRU. It first introduces a task-related representation vector as the benchmark for feature selection, which is called query vector. Then a scoring function is selected to calculate the correlation between the input feature and the query vector, and the probability distribution of feature selection is obtained, which is called attention distribution. Finally, the feature information related to the task is filtered out according to the weighted average of the input features according to the attention distribution, where *α*_*ij*_ represents the attention distribution coefficient of the *i* output sequence to the *j* input sequence, and its value is determined by the hidden layer state of each input and the *i* − 1 output. The smaller the value, the smaller the influence as

(13) $$\begin{array}{c} \alpha_{ij}=\frac{\exp\left(e_{ij}\right)}{\sum_{k=1}^{T_{x}}\exp\left(e_{jk}\right)}\text{.} \end{array}$$

After *α*_*ij*_ is calculated, the attention distribution vector of the output at time *i* in the *T*_*x*_ input hidden layer states is obtained through the softmax function; that is, the weight of *c*_*i*_ is calculated a

(14) $$\begin{array}{c} e_{ij}=\alpha \left(s_{i-1},o_{j}\right)=v^{T}\;\tanh\;\left(w_{s}s_{i-1}+w_{o}o_{j}\right)\text{.} \end{array}$$

### 3.3. English Intelligent Translation Model of LSTM-SA

Expressing the input model through fixed dimensions will lead to different translation emphases. The research adopts the English intelligent translation model to integrate the SA mechanism and LSTM expressing the input model through fixed dimensions which will lead to different emphases in translation. The framework of the LSTM neural network model based on the SA mechanism is as follows. The framework mainly includes five parts: input, deep neural network, LSTM, SA, and output layer. The load forecasting method is expressed as the original vector in the model layer and input into the matrix for calculation as *X*=[*x*_1_, *x*_2_, *x*_3_, ...,*x*_*n*_]^*T*^. The one-dimensional convolution used in the deep neural network layer has the characteristics of strong data feature extraction ability and can effectively mine the relationship between various types of data. Therefore, this paper studies how to extract data features through the convolution layer of deep neural network and introduces multisize convolution to make up for the disadvantage that the fixed convolution core cannot obtain more information. Finally, the model uses multiple convolution checks with different sizes to obtain multiple types of local features. Three convolution parallel structures are constructed in the deep neural network structure. After the data are input into the pooling layer, the model stores more data information through the maximum pooling method, realizes the maximum feature extraction of each vector, and splices the processed data to obtain a new vector to further obtain the maximum feature in the data [23]. Finally, input the connection layer, connect the data features extracted from the pooling layer, and then input them into the LSTM. Input vector *H*_*c*_ is calculated as

(15) $$\begin{array}{c} \left\{\begin{array}{c} C_{1}=f\left(X⊗W_{1}+b_{11}\right),C_{2}=f\left(X⊗W_{2}+b_{12}\right),C_{3}=f\left(X⊗W_{3}+b_{13}\right),\\ P_{1}=\max\left(C_{1}\right)+b_{21},P_{2}=\max\left(C_{2}\right)+b_{22},P_{3}=\max\left(C_{3}\right)+b_{23},\\ Hc=P_{1}+P_{2}+P_{3}. \end{array}\right. \end{array}$$

In formula (15), *P*_1_, *P*_2_, and *P*_3_ represent the output of the pool layer; *C*_1_, *C*_2_, and *C*_3_ indicate the output of convolution layer; *W*_1_, *W*_2_, and *W*_2_ represent the weight matrix; *b*_11_, *b*_12_, *b*_13_, *b*_21_, *b*_22_, *b*_23_ represent deviation; max () represents the maximum function value; and ⊗ represents convolution operation.

The data learned by LSTM is imported into the three SA mechanisms, and this kind of information is deeply mined, which enhances the attention of key information and improves the feature vector of load data [24]. At the same time, the dropout layer is introduced into the connection layer of the SA mechanism to avoid over fitting. The dropout layer can effectively ignore some nodes and prevent excessive dependence on eigenvalues in the process of model training.

The English intelligent translation model constructed by the research is shown in Figure 3. Firstly, calculate the correlation between key elements and a certain element, obtain the similarity, then standardize the similarity between them, then calculate the characteristic weight coefficient, and finally calculate the weighted sum weight vector. In the prediction process of the model, when the three mechanisms are equal, input a section of data, and then calculate the SA weight of each data point and other data points in the section of data. After adding the self-attention mechanism to the model, the ability of the model to capture medium and long-distance dependence features is improved. Because any two data can calculate the results through the weight matrix of the self-attention model and connect the results, the relationship between distance dependent features is shortened. The data learned by LSTM is imported into the three SA mechanisms, and this kind of information is deeply mined, which enhances the attention of key information and improves the feature vector of load data. At the same time, the dropout layer is introduced into the connection layer of the SA mechanism to avoid over fitting. The dropout layer can effectively ignore some nodes and prevent excessive dependence on eigenvalues in the process of model training. The output layer reduces the dimension of the input data by the characteristics of the full connection layer and outputs it.

## 4. Application Effect Analysis of English Intelligent Translation

The experiment analyzes the effect of English intelligent translation application through simulation experiments. The LSTM parameters are set as follows: dropt is 0.5, batch size is 128, the number of LSTM network layers is 2, the number of hidden layer and word vector nodes is 512, and the vocabulary is 30000. The dataset used in the experiment is the data of the 2020 International Oral and Translation Evaluation Competition, including 1 pair of development data, 3 pairs of test set data, and 220000 Chinese English parallel sentences.  Figure 4 shows the training loss results of common deep learning neural networks. As a whole, it can be seen that the training loss values of the four network structures continue to decrease with the increase of the number of iterations. The loss value of gate recurrent unit (GRU) and RNN is higher than that of LSTM and LSTM-SA. Both LSTM and LSTM-SA neural network algorithms converge rapidly when the number of iterations is about 20, and the gap between the two algorithms is not particularly obvious.

Figure 5 shows the network structure accuracy of LSTM neural network under different learning rates. When the ratio of LSTM neural network is 1/2, 1, and 2 respectively, the corresponding optimal regional scales are 3.7, 3.6, and 3.5, and the accuracy is 98.9%, 87.1%, and 89.5%, respectively.

Figure 6shows the network structure accuracy of LSTM-SA neural network under different learning rates. It can be seen that when the adaptability of LSTM-SA neural grid is 1/2, 1, and 2, respectively, the corresponding optimal regional scales are 4.4, 3.7, and 3.4, and the accuracy is 71.9%, 81.1%, and 71.9%, respectively. The accuracy of LSTM-SA neural network structure improved the fastest, and the accuracy improved by nearly 20%. When the adaptive degree is 1, the accuracy of the two structures has little difference, and the maximum accuracy difference is only 6.0%.

The experiment detects the effect in English intelligent translation through the loss value judgment model and uses the tensor board to show the change trend of loss. By introducing the attention mechanism of uncertainty loss function, the problem of subjectively setting main tasks and auxiliary tasks in the study of multilingual translation detection is solved. The model can still get ideal solution without dividing the main task and the auxiliary task. The loss results of content and noise are shown in Figures 7(a) and 7(b), respectively. The model loss value is to evaluate the effect of English intelligent translation from a quantitative perspective. The style loss and overall loss decreased gradually with the increase of training times, and the loss value quickly reached the convergence value, which were 0 and 2.000 *e* + 6, respectively.

The style and overall loss results are shown in Figures 8(a) and 8(b), respectively. The overall loss value is to evaluate the effect of English intelligent translation from a quantitative perspective. The style loss and overall loss decreased gradually with the increase of training times, and the loss value quickly reached the convergence value, which were 0 and 2.000 *e* + 6, respectively. The noise loss curve first rises rapidly and then converges slowly, and the existence value of convergence is repetitive, and the loss peak is 6.6 *e* + 4. The convergence speed of content loss is slow and can reach an optimal convergence value, and the loss value has a certain repeatability.

The number of hidden layers set in the experiment is 3, 5, and 7, respectively. The translation level map results of different depth learning algorithms are shown in Figure 9. Compared with other deep learning algorithms, the LSTM-SA neural network algorithm has a better translation level map under the three hidden layers. When the number of hidden layers is 3, 5, and 7, respectively, the translation levels map of LSTM-SA convolutional neural network are 74.3%, 73.8%, and 45.1%, respectively, and the translation levels map of LSTM convolutional neural network are 72.6%, 71.5%, and 42.1%, respectively, the translation levels map of RNN neural network are 71.1%, 70.6%, and 40.1%, respectively, and the translation levels map of GRU neural network are 67.5%, 65.0%, and 38.8%, respectively.

The experiment randomly selected six dimensions of English interest, English training times, vocabulary, sentence, content relevance, and relevance to evaluate the performance of three models. The six dimensions are represented by dimension 1–dimension 6 in turn. The accuracy and coverage are shown in Figure 10. On the whole, the accuracy difference of the six dimensions in the same model is not particularly large, but there are great differences in the accuracy of different models. There is a big gap in the coverage of the six dimensions in the same model and different models. It is worth noting that the accuracy of the six dimensions in the LSTM-SA model is higher, followed by LSTM and finally GRU. The accuracy rates of dimension 1–dimension 6 in the fusion model were 93.51%, 92.45%, 9037%, 92.36%, 91.81% and 92.15%, 88.07%, 86.23%, 90.73%, 84.82%, 89.32%, and 87.26% in the deep neural network model and 87.01%, 86.99%, 88.72%, 85.12%, 82.72%, and 86.25% in the linear regression model.

## 5. Conclusion

Aiming at the problems of poor translation quality in English intelligent translation, an English intelligent translation model based on LSTM-SA is proposed, and its performance is compared with other deep neural network models. The results show that the loss values of LSTM-SA, LSTM, RNN, and GRU neural network algorithms have the same trend in the first 20 generations of iterations, but in the range of 20 ∼ 100 iterations, the LSTM-SA neural network algorithm has faster convergence speed and more stable loss values. The action detection results of LSTM-SA and LSTM neural network structures show that when the adaptability of neural grid is 1/2, 1, and 2, respectively, and the optimal regional scale of LSTM-SA neural network is 4.4, 3.7, and 3.4, and the accuracy is 71.9%, 81.1%, and 71.9% respectively. The optimal regional scale of LSTM convolution neural network structure is 3.7, 3.6, and 3.5 and the accuracy is 98.9%, 87.1%, and 89.5%, respectively. The style loss and overall loss decreased gradually with the increase of training times, and the convergence values were 0 and 2.000 *e* + 6, respectively. The noise loss curve first rises rapidly and then converges slowly, and the existence value of convergence is repetitive, and the loss peak is 6.6 *e* + 4. When the number of hidden layers is 3, 5, and 7, the translation level map of LSTM-SA neural network is 74.3%, 73.8%, and 45.1%, respectively, and the corresponding values are better than the other three deep learning algorithms. The accuracy difference of the six dimensions in the same model is about 3%, while the accuracy difference in different models is less than 8%. Limited by my time and energy, there are still some problems in the research. In the follow-up, it is necessary to further optimize the network structure and improve the detection accuracy of English intelligent translation.

## Figures and Tables

**Figure 1:** Schematic diagram of the LSTM neural network structure.

**Figure 2:** Basic structure of the attention mechanism.

**Figure 3:** LSTM model framework based on the SA mechanism.

**Figure 4:** Training loss results of common deep learning algorithms.

**Figure 5:** Structure accuracy of LSTM convolutional neural network.

**Figure 6:** Structure accuracy of LSTM-SA convolutional neural network.

**Figure 7:** Contents and noise loss results. (a) Content image loss results. (b) Noise image loss results.

**Figure 8:** Style and overall loss results. (a) Style loss results. (b) Total loss result.

**Figure 9:** Translation level map results of different depth learning algorithms.

**Figure 10:** Accuracy evaluation results of three models.

## Data Availability

The data used to support the findings of this study are available from the corresponding author upon request.
